# Silencing of SOX12 by shRNA suppresses migration, invasion and proliferation of breast cancer cells

This article has been retracted.

**DOI:** 10.1042/BSR20160053

**Published:** 2016-10-06

**Authors:** Hanzhi Ding, Hong Quan, Weiguo Yan, Jing Han

**Affiliations:** * Department of Breast Surgery, Shanghai East Hospital, Tongji University School of Medicine, Shanghai 200120, China

**Keywords:** breast cancer, cell cycle arrest, invasion, migration, proliferation, SOX12

## Abstract

Sex determining region Y-box protein 12 (SOX12) is essential for embryonic development and cell-fate determination. The role of SOX12 in tumorigenesis of breast cancer is not well-understood. Here, we found that SOX12 mRNA expression was up-regulated in human breast cancer tissues. To clarify the roles of SOX12 in breast cancer, we used lentiviral shRNAs to suppress its expression in two breast cancer cells with relatively higher expression of SOX12 (BT474 and MCF-7). Our findings strongly suggested that SOX12 was critical for cell migration and invasion of breast cancer cells. We found that silencing of SOX12 significantly decreased the mRNA and protein levels of MMP9 and Twist, while notably increased E-cadherin. Moreover, SOX12 knockdown significantly inhibited the proliferation of breast cancer cells *in vitro* and the growth of xenograft tumours *in vivo*. Flow cytometry analysis revealed that breast cancer cells with SOX12 knockdown showed cell cycle arrest and decreased mRNA and protein levels of proliferating cell nuclear antigen (PCNA), CDK2 and Cyclin D1. Taken together, SOX12 plays an important role in growth inhibition through cell-cycle arrest, as well as migration and invasion of breast cancer cells.

## Abstract (precis)

SOX12 mRNA expression was up-regulated in human breast cancer tissues. SOX12 was critical for cell migration, invasion and proliferation of breast cancer cells.

## INTRODUCTION

Breast cancer is one of the most common and important malignant tumours affecting women. Despite the advances in screening, prevention, surgical resection and adjuvant therapies, breast cancer still remains the leading cause of death in women worldwide, accounting 23% of all cancer deaths [1]. Metastasis of breast cancer to other organs is the major cause of breast cancer deaths [2,3]. Consequently, there is a disquieting need to identify novel diagnosing marker and effective therapeutic targets for breast cancer.

Sex determining region Y-box protein 12 (SOX12) is a member of SOX genes, which encode a family of transcription factors belonging to the high mobility group (HMG) superfamily. SOX family proteins are important for embryonic developmental processes [4]. Disruption of SOX genes has been involved in various human diseases including cancer [5,6]. SOX family members may act as oncogenes or tumour suppressor genes. It is reported that SOX2 [7,8], SOX5 [9–11], SOX9 [12–14] and SOX18 [15] act as oncogenes in multiple types of human cancers through promoting cell proliferation, migration and invasion. On the contrast, SOX1 [16], SOX6 [17] and SOX7 [18,19] serves as a tumour suppressor gene to suppress cell proliferation and metastasis. A previous study has reported the critical role of SOX12 in embryonic development and cell-fate determination [20]. Recently, Huang et al. [21] demonstrated that SOX12 can promote invasion and metastasis of hepatocellular carcinoma (HCC). However, the expression and function of SOX12 in breast cancer remains unknown.

In this work, we presented the first evidence that SOX12 was overexpressed in breast cancer. We also investigated the potential role of SOX12 in breast cancer by knocking down its expression in two breast cancer cell lines. SOX12 knockdown inhibited migration and invasion of breast cancer cells. SOX12 knockdown also suppressed cell proliferation *in vitro* and growth of xenograft breast tumours *in vivo*. Together, our data strongly suggest the important role of SOX12 in the tumorigenesis and development of breast cancer.

## MATERIALS AND METHODS

### Patient samples

From June 2009 to July 2010, 35 patients with breast cancer (6 in AJCC stage I, 20 in stage II and 9 in stage III) admitted to Department of Breast Surgery, Shanghai East Hospital (Shanghai, China) with written informed consent were selected in this study. The patients had not received chemotherapy or radiation before surgery. The median age of the participants was 58 years (ranging from 35 to 78 years). The diagnosis of each case was independently confirmed by two pathologists. Human breast cancer and paired normal adjacent tissues (>2 cm from cancer tissue) were resected, snap frozen and then stored at -80°C until further use. This study was approved by the ethics committee of Shanghai East Hospital (Shanghai, China).

### Cell culture

HEK-293T and human breast cancer cell lines, MDA-MB-231, MCF-7, SK-BR-3, BT474, ZR-75-1 and ZR-75-30 were obtained from A.T.C.C. All cells were maintained in Dulbecco's minimum essential medium (DMEM) (Life Technologies) supplemented with 10% FBS (Hyclone), 100 units/ml penicillin and 100 μg/ml streptomycin at 37°C in a 5% CO_2_ atmosphere.

### RNA preparation and real-time PCR

Total RNA was prepared from the tissue samples or breast cancer cell lines by using TRIzol reagent (Invitrogen). First-strand cDNA was synthesized from total RNA with the M-MLV reverse transcriptase (Promega) following the manufacturer's manual. Quantitative real-time PCR was performed using the SYBR Green mix (Thermo Fisher Scientific) on the ABI Prism 7300 sequence detection system (Applied Biosystems). Primer sequences were 5’-AGCACCCGTGTGACTCTTTCC-3’ and 5’-AGCAGAACCAAGCCCTGTCTC-3’ for *SOX12*; 5’-AAGGGCGTCGTGGTTCCAACTC-3’ and 5’-AGCATTGCCGTCCTGGGTGTAG-3’ for *MMP9*; 5’-AGTCCGCAGTCTTACGAG-3’ and 5’-GCTTGCCATCTTGGAGTC-3’ for Twist1; 5’-GAGAACGCATTGCCACATACAC-3’ and 5’-AAGAGCACCTTCCATGACAGAC-3’ for E-cadherin; 5’-GGTGTTGGAGGCACTCAAGG-3’ and 5’-CAGGGTGAGCTGCACCAAAG-3’ for PCNA; 5’-AACAAGTTGACGGGAGAG-3’ and 5’-AAGAGGAATGCCAGTGAG-3’ for CDK2; 5’-GCTGCGAAGTGGAAACCATC-3’ and 5’-CCTCCTTCTGCACACATTTGAA-3’ for Cyclin D1; 5’-CACCCACTCCTCCACCTTTG-3’ and 5’-CCACCACCCTGTTGCTGTAG-3’ for *GAPDH*. The relative expression of the genes was calculated using the comparative cycle threshold (*C*_T_) method (2^ − Δ*C*_T_^) [22].

### shRNA constructs and lentiviral infections

For SOX12 knockdown, pLKO-1 plasmid containing shRNA-targeting targeting position 3728–3750 (GCTGCTTCACAGGATGAAA, shSOX12-1) and 4616–4638 (CAGGTGCTTATTCCTAATA, shSOX12-2) of human SOX12 and a non-specific scramble shRNA sequence (CCTAAGGTTAAGTCGCCCTCG, shNC) were constructed. The lentivirus particles were produced in HEK-293T cells transfected with psPAX2, PMD2G (Addgene) and pLKO-shRNA-containing plasmids. BT474 cells were infected with the lentivirus and stable cells were established by puromycin selection (Sigma).

### Western blotting and quantification

Cells were lysed in RIPA Lysis buffer [50 mM Tris/HCl, pH 8.0, 250 mM NaCl, 1% NP40, 0.5% (w/v) sodium deoxycholate, 0.1% sodium dodecylsulfate] supplemented with protease inhibitors (Roche). Whole-cell extracts containing 40 μg protein were electrophoresed on sodium dodecyl sulfate polyacrylamide (SDS-PAGE) gels, then transferred to polyvinylidene difluoride membranes (Millipore) and blocked in TBST-T with 5% skim milk. Anti-E-cadherin, proliferating cell nuclear antigen (PCNA), CDK2, Cyclin D1 and anti-GAPDH (Cell Signaling Technology) were used at 1:1000 dilution with overnight incubation at 4°C in TBS-T with 5% BSA. Anti-SOX12, Twist and MMP9 antibodies (Abcam) were used at 1:1000 dilution. After incubation with a horseradish peroxidase (HRP)-linked secondary antibody (Beyotime), blots were detected with Clarity Western ECL kit (Bio-Rad Laboratories). Band intensities were quantified by using ImageJ software (http://rsb.info.nih.gov/ij/).

### Transwell assay

Effect of SOX12 knockdown on cell motility and invasion were quantified by Transwell chamber (Costar). For cell invasion assay, the filters were pre-coated with Matrigel. Briefly, BT474 or MCF-7 cells were infected with shSOX12-1, shSOX12-2 or shNC virus and cultured at 37°C for 24 h. After starving in FBS-free DMEM medium overnight, cells in in serum-free medium were added into 24-well inserts (2×10^4^ cells per well). DMEM medium containing 10% FBS was added to the lower well of the chambers as chemoattractant. After 24 h, the cells on the upper surface of the filter were completely removed and migrated cells were fixed with 4% paraformaldehyde and stained with 0.5% crystal violet. Cells traversing the membrane were counted in 10 random fields under a microscope.

### Cell proliferation assays

Effect of SOX12 knockdown on cell proliferation was measured by using CCK-8 (Dojindo Laboratories). Briefly, BT474 or MCF-7 cells were plated on to 96-well plates at density of 3×10^3^ cells per well. After cultured overnight, cells were infected with the shSOX12-1, shSOX12-2 virus or control virus (shNC). At 0 h, 24 h, 48 h and 72 h after viral infection, CCK-8 solution was added to every well and incubated at 37°C for 1 h. Absorbance (*A*) values were determined at wavelength 450 nm (*A*_450_) on a microplate reader (Bio-Rad Laboratories).

### Tumour xenografts

Four to five-week-old female BALB/c nude mice were purchased from Shanghai Laboratory Animal Company and maintained under standard conditions in line with the NIH Guide for the Care and Use of Laboratory Animals. BT474 cells stably infected with shNC or shSOX12-1 were collected, resuspended in PBS and injected subcutaneously into the right flank of each mouse (2×10^4^ per mouse). Tumour xenografts were measured with calipers every 3 days, and tumour volume was determined using the following formula: (length × width^2^) × 0.5. At the end of the experiment, after anesthetized with sodium pentobarbital, the mice were killed by cervical dislocation and tumour xenografts were recovered. A portion of tissues were fixed in formalin, processed to obtain sections of 5 μm and stained with using haematoxylin and eosin (HE) or PCNA (Abcam) immunohistochemically. The other portion of tissues was employed for protein extraction and Western blotting analysis to examine SOX12 expression. All experiments were approved by the Committee on the Ethics of Animal Experiments of Shanghai East Hospital (Shanghai, China).

### FACS analysis

BT474 or MCF-7 cells were infected with shSOX12-1, shSOX12-2 or shNC virus and cell cycle distribution was monitored 48 h after viral infection. The cells were collected, washed with PBS and fixed in ice-cold ethanol at -20°C overnight. The cells were washed with PBS and resuspended in PBS buffer containing RNase A (1 mg/ml, Sigma) at 37°C for 30 min. The cells were then stained with propidium iodide (PI, 60 μg/ml, Sigma) and analysed for DNA content with a flow cytometer (Accuri C6, BD).

### Statistics

All statistics were calculated using GraphPad Prism, version 6.0 (GraphPad). All *in vitro* experiments assays were performed in triplicate, and mean values and S.D. were reported. Differences between groups were determined by Student's *t* test. *P*   less than 0.05 was considered statistically significant.

## RESULTS

### *SOX12* is overexpressed in breast cancer compared with normal breast tissue

To assess SOX12 expression in breast cancer, real-time RT-PCR was used to evaluate SOX12 expression level in 35 breast cancer tissues and paired normal tissues. As shown in Figure 1, SOX12 expression was significantly increased in 94% (33/35) of breast cancer tissues when compared with normal tissues.

**Figure 1:** SOX12 is overexpressed in breast cancer. Real-time PCR analysis of SOX12 mRNA levels in 35 pairs of breast cancer and normal tissues. Positive log 2 (Tumour/Normal) on the *y*-axis indicated the elevated expression of SOX12 in tumour tissue whereas negative log 2 indicated the reduced expression of SOX12 in tumour tissue.

### Knockdown of SOX12 in breast cancer cells

To investigate the role of SOX12 in breast cancer, the mRNA levels of SOX12 were evaluated in six human breast cancer cell lines, including MDA-MB-231, MCF-7, SK-BR-3, BT474, ZR-75-1 and ZR-75-30, by performing real-time PCR analysis (Figure 2A). The expression levels of SOX12 were much higher in MCF-7 and BT474 cells than in other four cell lines. The higher expression level of SOX12 was confirmed at the protein level by Western blot analysis in both MCF-7 and BT474 cells (Figure 2B), which were selected for the following experiments.

**Figure 2:** Knockdown of SOX12 in breast cancer cells. (**A**) The mRNA expression levels of SOX12 in six human breast cancer cells were determined by real-time PCR and normalized with GAPDH. (**B**) The protein levels of SOX12 were determined in human breast cancer cells by Western blot. GAPDH was used as the loading control. (**C**) Knockdown of SOX12 in BT474 and MCF-7 cells detected by real-time PCR. (**D**) Knockdown of SOX12 in BT474 and MCF-7 cells detected by Western blot. Upper panels: representative images; lower panels: quantifications of Western blot. WT: wild-type cells; shNC: cells infected with scrambled shRNA virus; shSOX12-1: cells infected with shSOX12-1 virus; shSOX12-2: cells infected with shSOX12 virus. **P<0.01 and ***P<0.001 compared with shNC.

To study the role of SOX12 on breast tumorigenesis, SOX12-shRNA lentivirus (shSOX12-1 and shSOX12-2) and non-specific scramble shRNA lentivirus (shNC) were produced and infected BT474 and MCF-7 cells, which have high endogenous SOX12 levels. At 48 h after lentiviral infection, mRNA and protein levels of SOX12 were measured. As shown in Figures 2(C) and 2(D), shSOX12 viral infection significantly decreased SOX12 expression at both mRNA and protein levels compared with those of wild-type (WT) and shNC lentivirus infected cells.

### SOX12 knockdown inhibits migration and invasion of breast cancer cells

Huang et al. [21] have demonstrated the promoted effects of SOX12 on the invasion and metastasis of HCC. To investigate the effects of SOX12 on the invasion and migration capacities of breast cancer cells, Transwell assays were performed. As shown in Figures 3(A) and 3(B), infection with shSOX12-1 and shSOX12-2 virus in both BT474 and MCF-7 cells notably reduced the abilities of invasion and migration compared with WT and shNC cells, whereas no significant difference was observed in the invasive capability between WT and NC cells. In addition, protein levels of epithelial–mesenchymal transition (EMT)-related proteins, which contribute to metastasis of tumour cells, were evaluated by Western blot. Infection with shSOX12-1 and shSOX12-2 virus significantly decreased the protein levels of MMP9 and Twist, while notably increased the main factor of EMT, E-cadherin (Figures 3C and 3D). These results demonstrated that SOX12 promoted the abilities of invasion and migration of breast cancer cells.

**Figure 3:** SOX12 knockdown inhibited the migration and invasion ability of breast cancer cells. (**A**) SOX12 knockdown inhibited the migration ability of BT474 and MCF-7 cells as determined by Transwell assays in chambers without Matrigel. Left panels: representative images; right panels: quantifications of average migrated cell number. (**B**) SOX12 knockdown repressed the invasion ability of BT474 and MCF-7 cells as determined by Transwell assays in chambers coated with Matrigel. Left panels: representative images; right panels: quantifications of average migrated cell number. (**C** and **D**) The levels of MMP9, Twist and E-cadherin were examined with real-time PCR and Western blot. GAPDH was used as internal control. Left panels: real-time PCR results; middle panels: representative images of Western blot; right panels: quantifications of Western blot. WT: wild-type cells; shNC: cells infected with scrambled shRNA virus; shSOX12-1: cells infected with shSOX12-1 virus; shSOX12-2: cells infected with shSOX12 virus. *P<0.05, **P<0.01 and ***P<0.001 compared with shNC.

### Knockdown of SOX12 suppresses the proliferation of breast cancer cells *in vitro* and *in vivo*

In addition to promoting metastasis, we investigate the effect of SOX12 on cell proliferation in breast cancer cells by CCK-8 assay. Knockdown of endogenous SOX12 significantly inhibited the growth of BT474 cells (Figure 4A) and MCF-7 (Figure 4B) at 24 h, 48 h and 72 h after viral infection. Consistent with the results obtained from *in vitro* assays, knockdown of endogenous SOX12 reduced the growth of BT474 xenograft tumours (Figures 4C and 4D). Protein levels of SOX12 were significantly lower in the xenografts formed from shSOX12-1 stable cells than in those from shNC stable cells (Figure 4E). Further, immunohistochemical staining revealed that the PCNA-positive cells were significantly reduced in the xenografts formed from shSOX12-1 stable cells compared with those from shNC cells (Figure 4F). Together, these results demonstrated that SOX12 shRNA inhibited the proliferation of breast cancer cells and the growth of xenograft breast tumours.

**Figure 4:** Knockdown of SOX12 suppressed the proliferation of breast cancer cells *in vitro* and *in vivo.* (**A** and **B**) Knockdown of endogenous SOX12 inhibited the growth of BT474 and MCF-7 cells. (**C**–**F**) SOX12 knockdown reduced the growth rate of xenograft breast tumours. BALB/c nude mice were inoculated with BT474 cells stably infected with shNC or shSOX12 virus (*n*=6). The tumour size was monitored every 3 days and growth curves of xenograft tumours were shown in (**C**). At 33 days after inoculation, the mice were killed and the tumours were recovered. Images of and weights of xenograft tumours were shown in (**D**). The expression of SOX12 in xenograft from the nude mice was determined by Western blot (**E**). Representative images of HE staining and PCNA immunohistochemical staining of xenograft tumours were shown in (**F**). **P<0.01 and ***P<0.001 compared with shNC.

### Knockdown of SOX12 induces G1-arrest in breast cancer cell lines

Then we assessed the effect of SOX12 on the cell cycle of breast cancer cells by flow cytometry analysis. The results show that infection with shSOX12-1 virus caused an accumulation of BT474 and MCF-7 cells at the G0/G1 phase, whereas the percentages of cells in S phase and G2/M phase decreased (Figures 5A and 5B). Moreover, the protein levels of G1/S transition-related proteins were also evaluated by Western blot. Infection with shSOX12-1 virus significantly decreased the protein levels of PCNA, CDK2 and Cyclin D1 (Figures 5C and 5D). These results indicated that SOX12 knockdown contributed to induction of G1-arrest in breast cancer cells.

**Figure 5:** SOX12 knockdown induced G1 arrest. BT474 and MCF-7 cells were infected with shSOX12 or shNC virus. (**A** and **B**) At 48 h after viral infection, cell cycle distribution of BT474 and MCF-7 cells infected with shSOX12 or shNC virus. (**C** and **D**) At 48 h after viral infection, the levels of PCNA, CDK2 and Cyclin D1 were examined with Western blot. GAPDH was used as the loading control. Left panels: real-time PCR results; middle panels: representative images of Western blot; right panels: quantifications of Western blot. WT: wild-type cells; shNC: cells infected with scrambled shRNA virus; shSOX12: cells infected with shSOX12 virus. **P<0.01 and ***P<0.001 compared with shNC.

## DISCUSSION

SOX12 plays an essential role in embryonic development and cell-fate determination [20]. A recent study has suggested SOX12 may play a role in the tumorigenesis of HCC [21], whereas the association between SOX12 and breast cancer has not been reported. Our results showed that SOX12 mRNA expression was elevated in breast cancer tissues (Figure 1), suggesting that SOX12 may also serve as an oncogene in breast cancer.

Metastasis to vital organs is the major cause of mortality from breast cancer [2,3]. Cell migration and invasion are indispensable processes for the metastasis of cancer. In the present study, Transwell assays showed that SOX12 contributed to breast cancer cell migration and invasion, as a reduction in SOX12 protein by RNAi caused significant decreases in the migration and invasion of BT474 and MCF-7 cells (Figures 3A and 3B). Further, the EMT is implicated in promoting carcinoma invasion and metastasis [23,24]. Here, shSOX12 viral infection enhanced the expression of the main factor of EMT (E-cadherin [25]), but decreased the expression of a known inducer of EMT (Twist [26]) (Figures 3C and 3D). The mRNA levels of E-cadherin and Twist were also changed after SOX12 knockdown, indicating that SOX12 may bind to the promoters of these EMT-regulating factors to control their transcription. It has been reported that SOX12 promotes migration and invasion of HCC through up-regulating Twist1 and FGFBP1 [21]. Together with the study on HCC, our data suggested that SOX12 may prompt cell invasion through inducing EMT.

Previous studies have shown the role of other members of SOX family in the proliferation of tumour cells [12,15,16,19]. Results from the current study demonstrated that knockdown of SOX12 inhibited the proliferation of breast cancer cells *in vitro* and *in vivo* (Figure 4). Further, we demonstrated that shSOX12 viral infection significantly decreased mRNA and protein levels of PCNA, CDK2 and Cyclin D1. These results are consistent with the increased percentages of G1 phase shown in the shSOX12-infected cells (Figure 5). SOX12 may bind to the promoter regions of the above genes to influence their transcription, although further investigation is required to verify this hypothesis.

In summary, we revealed that SOX12 expression was up-regulated in breast cancer tissues. Moreover, we showed that SOX12 plays an important role in promoting growth, migration and invasion of breast cancer cells. This study suggested that SOX12 may be an important biomarker for breast cancer and may lead to new therapeutic approaches for breast cancer.

## Abbreviations

DMEM: Dulbecco's minimum essential medium
EMT: epithelial–mesenchymal transition
HCC: hepatocellular carcinoma
HE: haematoxylin and eosin
OD: optical density
PCNA: proliferating cell nuclear antigen
PI: propidium iodide
SOX12: sex determining region Y-box protein 12
WT: wild-type
